The article "Variant Analysis of Alkaptonuria Families with Significant Founder Effect in Jordan" was published in 2021. Journal: Biomed Res Int.

# Variant Analysis of Alkaptonuria Families with Significant Founder Effect in Jordan

**DOI:** 10.1155/2021/1515641

**Published:** 2021-03-11

**Authors:** Raida Khalil, Dema Ali, Nesrin Mwafi, Arwa Alsaraireh, Loiy Obeidat, Eman Albsoul, Ibrahim Al Sbou'

**Affiliations:** ^1^Department of Biotechnology and Genetic Engineering-Faculty of Science, University of Philadelphia, Amman, Jordan; ^2^Cell Therapy Center, The University of Jordan, Amman, Jordan; ^3^Department of Biochemistry and Molecular Biology, Faculty of Medicine, Mutah University, AlKarak, Jordan; ^4^Maternal and Child Health Nursing Department, Faculty of Nursing, Mutah University, AlKarak, Jordan; ^5^Medical Laboratory Science, Faculty of science, Mutah University, AlKarak, Jordan

## Abstract

**Background:**

Metabolic disorder alkaptonuria is an autosomal recessive disorder caused by mutations in the *HGD* gene, and a deficiency HGD enzyme activity results in an accumulation of homogentisic acid (HGA), ochronosis, and destruction of connective tissue.

**Methods:**

We clinically evaluated 18 alkaptonuria patients (age range, 3 to 60 years) from four unrelated families. Furthermore, 11 out of 18 alkaptonuria patients and 7 unaffected members were enrolled for molecular investigations by utilizing Sanger sequencing to identify variants of the 14 exons of *HGD* gene.

**Results:**

We found that the seven patients from the 4 unrelated families carried a recurrent pathogenic missense variant (c.365C>T, p. Ala122Val) in exon 6 of *HGD* gene. The variant was fully segregated with the disease in affected family members while the other unaffected family members were heterozygous carriers for this variant. Additionally, the clinical features were fully predicted with alkaptonuria disorder.

**Conclusion:**

In this study, we confirmed that the most common variants in Jordanian AKU patients was c.365C>T, p. Ala122Val in exon 6 of *HGD* gene. Additionally, we correlated the clinical and genetic features of AKU patients at various ages (3-60 years).

## 1. Introduction

Alkaptonuria (AKU) was first described by Garrod in 1908 as an inborn defect in metabolism (Garrod 1908). Alkaptonuria is a rare autosomal recessive disease with an estimated frequency of 1 : 250,000-1,000,000 among most ethnicities. The true prevalence of AKU might be underestimated due to the subtle signs of the disease, causing many patients to go throughout life undiagnosed [1, 2]. Several variants of the homogentisate 1,2-dioxygenase (*HGD*) gene have been reported as disease-causing variants. This gene is located on the long arm of chromosome 3 (q23-q21) and contains 14 exons. The HGD enzyme is the protein product of this gene and consists of 445 amino acids, with an expression pattern of protein localization to the kidney, liver, and cartilage [3–5]. The HGD enzyme plays a key role in the tyrosine catabolism pathway by converting homogentisic acid into maleylacetoacetic acid. Mutations in the *HGD* gene result in an inactive form of the enzyme, which results in the accumulation of homogentisic acid [6]. Part of the generated homogentisic acid is cleared by the kidneys, which darkens the urine colour on standing or when it is treated with alkali [7, 8]. The remaining circulating homogentisic acid is distributed via the blood to various collagenous tissues and body fluids [9]. However, the interaction of homogentisic acid and its oxidation products with the connective tissue of affected individuals leads to severe arthritis, particularly in the spine and large joints, and might also lead to the destruction of the cardiac valve in severe cases [10].

The concentration of homogentisic acid in urine can be measured by gas chromatography and mass spectrometry analysis and serves as a quick diagnostic marker [11]. However, molecular genetic testing is critical to detect affected individuals and carriers of the disease. AKU pathology does not impact longevity in patients but significantly affects their quality of life. To date, no medication is approved to treat alkaptonuria, and patient life style must be adjusted to slow and manage disease symptoms [10]. HGA homopolymer deposition within the hyaline articular cartilage causes the associated joints to be weak and prone to rapid degeneration; hence, patients should not carry heavy objects that might harm the joints. In addition, adjusting nutritional habits to lower protein intake might reduce the levels of homogentisic acid and mitigate its negative impacts on the health of patients with AKU [12].

The most interesting aspect of the genetics of alkaptonuria is the heterogeneity of the *HGD* mutation among populations. Approximately 178 *HGD* variants affecting enzyme function have been identified and are reported in the *HGD* mutation database http://hgddatabase.cvtisr.sk. Missense substitutions account for 65% of the reported mutations. However, splice site mutations, deletions, duplications, and nonsense mutations have also been identified. Some mutations have been reported to be more prevalent among some populations than others [13, 14]. The missense G161R mutation occurring in exon 8 is the most prevalent in Slovakia, whereas M368V in exon 13 occurs among Europeans [14, 15]. So far, there are four HGD gene variants reported in Jordanian AKU patients: c.365C>T [14, 16], c.16-1G> [14, 17], c.16-272_c.87+305del, and c.87+8_88-31del765 [17].

Understanding the molecular basis of genetic diseases is of critical importance for the prevention of recurrence in future offspring and for the elucidation of disease mechanisms, which will aid the development of potential therapies.

The aims of this study were to conduct a mutational analysis of the *HGD* gene in families diagnosed with AKU and to provide information regarding the mutational background of Jordanian patients with AKU. For these purposes, Sanger sequencing was utilized as the main genetic analysis tool to screen the 14 exons of the homogentisate 1,2-dioxygenase gene in affected individuals.

## 2. Methods

### 2.1. Patients and Clinical Investigation

The current study was approved by the ethics committee in Mutah University, Jordan (No. 201955) and in accordance with the Helsinki Declaration of 1964. Informed consent was obtained from all participants involved in this study. We analysed 4 families from South Jordan for HGD gene variants. Eighteen patients with AKU were enrolled in the clinical study and ranged in age from 3 to 60 years old. Diagnoses of AKU were based on documented elevated homogentisic acid in urine (dark urine); bluish discoloration of the ear cartilage and teeth pigmentation (ochronosis); presence of renal stones; low back, shoulder, knee, and hip pain (ochronotic arthropathy); morning stiffness and swelling of small joints.

### 2.2. DNA Extraction

Peripheral blood samples for Sanger sequencing were collected from four unrelated families with AKU; samples were obtained from both patients with AKU (*N* = 11) and unaffected members (*N* = 7). Genomic DNA was extracted from whole blood using the G-spin™ Total DNA Extraction Mini Kit (iNtRON, Korea) according to the manufacturer's instructions. The quantity and quality of extracted DNA were measured by NanoDrop 2000 spectrophotometer (Thermo Fisher Scientific, USA).

### 2.3. Sanger Sequencing

Sanger sequencing was used to identify variants of the *HGD* gene. Seven probands from four selected families were tested for the 14 exons (coding regions) and intron-exon boundaries of the *HGD* gene. For the segregation analysis, other affected (*N* = 4) and unaffected members (*N* = 7) from the tested families were analysed for candidate variants. Briefly, PCR amplification was carried out using Phusion High-Fidelity PCR Master Mix (Thermo Fisher, USA) and specific primer pairs (Table 1). PCR products were separated on 2% gel and then purified with ExoSAP-IT™ PCR Product Cleanup Reagent (Applied Biosystems, USA). The purified PCR products were sent to Macrogen Sequencing Service (Macrogen, Korea) for sequencing. Sequence data were analysed with Chromas Pro software (Technolysium Ltd., South Brisbane, Australia). The effects of missense variants identified in the coding regions were predicted using in silico tools (PolyPhen2 http://genetics.bwh.harvard.edu/pph2/, SIFT http://sift.jcvi.org/, Mutation taster http://www.mutationtaster.org/). Variants occurring with a frequency of ≥1% were classified as benign. The identified variants were queried in the ClinVar database (https://www.ncbi.nlm.nih.gov/clinvar/) and the *HGD* mutation database (http://hgddatabase.cvtisr.sk/home.php?select_db=HGD).

## 3. Results

### 3.1. Clinical Features

The clinical findings of the 18 patients with AKU are summarized in Table 2 and Figure 1. Thirteen males and 5 females were registered in the current study (Table 2). The youngest patient was 3 years old, and the oldest was 60 years old. The most common clinical features were as follows: (1) dark urine (100%) (Figure 1(a)); (2) ear symptoms, including black ear wax (100%) (Figure 1(k)), bluish discoloration of ear cartilage (44%) (Figure 1(e)), and hearing impairments (33%); (3) brown spots in eye sclera (11%) (Figure 1(b)); (4) pigmentation of the teeth (44%) (Figure 1(c)); (5) recurrent renal stones (28%) (Figure 1(h)); (6) ochronotic arthropathy of the spine (56%) (Figure 1(j)), shoulder (28%) (Figure 1(f)), knee (22%), or hip (33%); (7) morning stiffness and low back pain (55%); (8) replacement of shoulder joint (5.5%); (9) Achilles tendon rupture (11%) (Figure 1(g)); (10) foot pain and swelling of interphalangeal joints (17%); and (11) skin pigmentation (11%) (Figures 1(d) and 1(i)).

### 3.2. Variant and Segregation Analysis

The result of Sanger sequencing revealed that the seven patients from the 4 unrelated families carried a recurrent pathogenic missense variant in exon 6 (c.365C>T, p. Ala122Val). The variants were fully segregated with the disease in affected family members (*N* = 11) (Figures 2 and 3). However, the other unaffected members were heterozygous carriers for this variant. This missense variant was detected with an allele frequency of 0.0056% in the gnomAD database. Additionally, the variant was predicted to be deleterious, probably damaging and disease causing in the SIFT, PolyPhen2 and mutation taster analyses, respectively (Table 3). Another missense variant in exon 4 (c.240A>T, p. Gln80His) of the *HGD* gene was identified as homozygous in all seven probands. This missense variant (c.240A>T, p. Gln80His) was detected with an allele frequency of 74% in the gnomAD database and founded in the HGD database as a benign variant.

## 4. Discussion

Alkaptonuria affects 1 in 250,000 to 1 million people worldwide [1, 18]. However, some areas, such as Slovakia and the Dominican Republic, show a much higher prevalence than others [7]. Although the prevalence of AKU in the Araba population is not well studied, it is likely to be high due to the high percentage of consanguineous marriages in the region [19]. The current study is aimed at determining the prevalence of pathogenic variants in the Jordanian population, specifically, villages located in the south region of Jordan. In the current study, the prevalence of pathogenic variants in the *HGD* gene was 100%. All affected members of the 4 candidate families were found to have the same pathogenic variant (c.365C>T) first reported by Phornphutkul et al. (2002) and reported as the most common variant in Jordanian and Indian populations [14, 16, 18, 20]. However, none of the other identified variants reported before (c.16-1G>, c.16-272_c.87+305del, c.87+8_88-31del765) in Jordanian population were found among the recruited families in the current study. This pathogenic variant is a founder variant for the patients with AKU in this region of Jordan, maintained by frequent consanguineous mating. The identified pathogenic variant was in exon 6 of the HGD gene (c.365C>T, p. Ala122Val). This variant has been widely studied with respect to the functional and structural effectiveness of the HGD enzyme [17]. Additionally, a common polymorphism (c.240A>T, p. Gln80His) in exon 4 of the *HGD* gene was determined to be homozygous in all the affected patients.

The main clinical signs and symptoms AKU include darkening of urine on standing as a result of the accumulation of HGA and its oxidation products, arthritis of the spine and larger joints, and connective tissue ochronosis. In some patients, the diagnosis of AKU is made only after the individual seeks medical attention for chronic joint pain or after black articular cartilage is noted. In the present study, the former mentioned sign was observed in the adult patients, whereas ear wax was observed in both adult and paediatric patients. Furthermore, hearing impairments were diagnosed in 33% of the adult patients [21]. All the enrolled patients had dark urine on standing; since darkening may not occur for several hours after voiding, many patients never observe such abnormal colouration of their urine. This phenomenon partially explains the late onset of diagnosis in most of the patients in the present study. On the other hand, none of the patients with AKU had cognitive impairment or developmental delay, and many had a long-life span, since some patients had reached over 40 years old. Ochronotic arthritis, which is a manifestation of longstanding alkaptonuria, was predicted in the studied patients at the second decade, in particular, joint symptoms involving the spine. Knee, hip, and shoulder symptoms were predicted at the third decade. However, only one patient had undergone joint replacement by age 43 years. Additionally, low back pain was observed in the adult group at ages greater than 20 years. This finding is in agreement with a previous study [18].

The kidneys are responsible for discharging enormous quantities of HGA in patients with AKU, leading to diminished renal function and the formation of renal stones, which were observed in most patients greater than 20 years of age or in the adult age group. Consequently, the development of ochronosis of the spine is accelerated, as previously reported [22].

In summary, we confirmed that the most common variant in *HGD* gene; c.365C>T, p. Ala122Val occurred at high prevalence among Jordanian patients with AKU. There is a possibility of detecting other pathogenic variants if more samples are analysed. It would be of interest to extend this study to a larger population of patients with AKU in different areas in Jordan to determine whether they carry the founder variant (c.365C>T, p. Ala122Val) or other variants of the *HGD* gene. However, since the current study identified the founder pathogenic variant (c.365C>T, p. Ala122Val) in the *HGD* gene, carrier testing for at-risk relatives and prenatal molecular diagnosis for pregnancies at increased risk are possible.

## Figures and Tables

**Figure 1:** The clinical features appeared in the investigated AKU patients. (a) The urine is converted from yellow to dark brown upon overnight standing, (b) brown spot appears in the sclera of the eye, (c) dark pigmentation of the teeth, (d) blue-black papules and plaques with pitting along the line of transgradience of the thumb and index finger, (e) bluish discoloration of the external ear cartilages, (f) ochronosis of the cartilage that cover the head of the humerus bone which is removed during the shoulder joint replacement surgery, (g) Achilles tendon rupture, (h) black renal stones from AKU patient, (i) ochronosis of the face and cheeks, (j) multiple degenerative changes in the dorsal spine with narrowing and calcifications of the intervertebral disc space shown in CT scan, and (k) black colour of the ear wax.

**Figure 2:** Pedigrees of four unrelated families with alkaptonuria found to carry a variant in the *HGD* gene; c.365C>T, p. Ala 122 Val in exon 6.

**Figure 3:** Variants chromatograph for the identified variants in the *HGD* gene. (a) Pathogenic variant in exon 6 of the *HGD* gene; c.365C>T, p. Ala122Val. (b) Benign variant in exon 4 of the *HGD* gene; c.240A>T, p. Gln80His.

**Table 1:** Primer oligonucleotide sequences used in Sanger sequencing.

Exon	Primer sequence (5′-3′)	Amplicon size (bp)	Annealing temperature (°C)
1	F: GAGTTAGACAATTCTTTCAGC	418	51
	R: ATGAACAAAGGCAAGGGATG		
2	F: GCAATATCCAGCACTCTTCTGA	437	55
	R: CCCCTATGACTTGGGAAACC		
3	F: GGGGCAAGTCACATCAAAAG	415	53
	R: GCTGGCAGGAAGTTCATTCT		
4	F: TTGGCAGCATGGAAATAACC	516	54
	R: TTTGAGCAGAAAACAGACACACT		
5	F: AGCATGAAAAGCAGCATCAG	560	53
	R: ACGCAGGTGGTTTTGTCTCT		
6	F: GTCAGTAAATTCAGGCTCCTTAGA	521	57
	R: TCCATCCTCCCTTTTCTGTTT		
7	F: CGCTATTCTTTCATTCCCTCA	530	52
	R: GTCCAGAAGAGATGGGCAAA		
8	F: ACAAGTTCCTTGCCTGGTGA	439	53
	R: CTCAGATTCCCTCCTCGTTG		
9	F: CCAAGCAGCTCAACAAACAA	319	55
	R: AGTGAGACAGCGAAGGGAGA		
10	F: CTCTCTTCCCTTCCCCTCAC	551	57
	R: TTTGTAGTGCCGTAGTGGTATGA		
11	F: TCTCCCAAAGGACGGTAAAA	391	53
	R: CTCCCTCACCAAAGGACAAA		
12	F: CAGATCCCTACCCCAAACCT	600	56
	R: CACGAGCCAAATGAACCTCT		
13	F: TGCCAAGAATGCCAATATGA	478	60
	R: CCCTCTTTTGACTCTTCCTCTG		
14	F: ACCAGAGCCACAACTCAGG	576	55
	R: CTGCCAGGTTTGTCTCATCA		

**Table 2:** Main clinical manifestations observed in AKU patients involved in the current study. M: male; F: female.

Patients' ID (pedigree)	Age of diagnosis (years)	Age and gender of the AKU patient	Dark urine	Main AKU signs and symptoms appeared in the patient														
				Ear symptoms			Brown spots in eye sclera	Skin pigmentation	Pigmentation of the teeth	Recurrent renal stones	Ochronotic arthropathy				Morning stiffness and low back pain	Replacement of shoulder joints	Achilles tendon rupture	Foot pain and swelling of interphalangeal joints
				Black ear wax	Bluish discoloration of ear cartilage	Hearing impairments					Spine	Shoulder	Knee	Hip				
AKU_AII:3	40	51/M	+	+	+	+	-	-	+	+	+	-	-	+	+	-	-	-
AKU_AII:4	35	46/M	+	+	+	+	-	-	+	+	+	+	-	-	+	-	-	+
AKU_AIII:1	9	18/F	+	+	-	-	-	-	-	-	-	-	-	-	-	-	-	-
AKU_BII:2	42	52/F	+	+	-	-	-	-	-	-	+	-	-	-	+	-	-	-
AKU_BII:3	50	60/F	+	+	-	-	-	-	-	-	+	-	-	-	+	-	-	-
AKU_BIII:6	36	41/M	+	+	+	+	+	+	+	+	+	+	-	-	+	-	-	-
AKU_BIV:2	1	9/M	+	+	-	-	-	-	-	-	-	-	-	-	-	-	-	-
AKU_BIV:3	4	12/M	+	+	-	-	-	-	-	-	-	-	-	-	-	-	-	-
AKU_BIV:4	7	15/M	+	+	-	-	-	-	-	-	-	-	-	-	-	-	-	-
AKU_BIV:6	6	11/M	+	+	-	-	-	-	-	-	-	-	-	-	-	-	-	-
AKU_BIV:7	4	9/F	+	+	-	-	-	-	-	-	-	-	-	-	-	-	-	-
AKU_CII:3	41	44/M	+	+	+	-	-	-	+	-	+	+	+	+	+	-	+	-
AKU_CII:4	34	37/M	+	+	+	-	-	-	+	-	+	+	+	+	+	-	-	+
AKU_CIII:2	6	8/M	+	+	-	-	-	-	-	-	-	-	-	-	-	-	-	-
AKU_CIII:3	1	3/M	+	+	-	-	-	-	-	-	-	-	-	-	-	-	-	-
AKU_DII:1	33	43/M	+	+	+	+	-	+	+	+	+	+	+	+	+	+	-	-
AKU_DII:2	25	35/M	+	+	+	+	+	-	+	+	+	-	+	+	+	-	+	-
AKU_DII:3	22	32/M	+	+	+	+	-	-	+	-	+	-	-	+	+	-	-	+

**Table 3:** *HGD* variants founded in the tested families.

Variant _ ENST00000283871.10					ClinVar	dbSNP ID	Protein prediction			MAF gnomAD (%)
Exon	Chromosome location (GRCh37)	HGVS cDNA	HGVS aa	Variant effect			SIFT	PolyPhen-2	Mutation taster	
E6	3 : 120369690	c.365C>T	p.Ala122Val	Missense	Likely pathogenic	rs544956641	Deleterious	Probably damaging	Disease causing	0.005569
E4	3 : 120670469	c.240A>T	p. Gln80His	Missense	Benign	rs2255543	Tolerated	Benign	Polymor-phism	74

## Data Availability

All relevant data is available through this manuscript.
